This article has been retracted.

# Visual Sensor Image Deconstruction in Constructing Green Building Design Space Adjustment Construction Strategy

**DOI:** 10.1155/2022/9137171

**Published:** 2022-09-10

**Authors:** Xiumin Xia

**Affiliations:** Ningbotech University, Ningbo, Zhejiang 315000, China

## Abstract

Since the introduction of green design in China, the space adjustment of green building design has received great attention from architects. Because space adjustment is very important for the pre-construction of a green building, it also represents the effectiveness of the building after its operation. At the same time, the spatial adjustment of green buildings is also a professional level test for architects. In order to obtain more accurate information about various aspects of the building, it is not enough to rely on the naked eye or measuring tools. Because it is impossible to comprehensively inspect the entire building, and the data is too cluttered, it is inconvenient to carry out a one-step construction strategy. Therefore, this study proposes to use visual sensors to analyze the image of a building, so as to achieve the data effect that architects want and to achieve the best effect in space adjustment. In order to prove the applicability of visual sensors, this study takes the current situation of domestic green building projects as a case study and deeply explores the status of domestic green building projects under the current social background. Then, the method of the visual sensor is used to analyze the problem of building space adjustment, and experimental research on the performance of this technology is carried out. The results show that this technology is very suitable for the study of construction strategies for spatial adjustment. In building identification, the error of the algorithm in this study in the measurement range of 1 m to 2 m is obviously smaller than that of other methods, and the accuracy is basically kept within 1 cm. Therefore, in order to better develop the green design, we should focus on the application of visual sensors in this regard.

## 1. Introduction

The concept of green design is to save resources and protect the environment, which is now the most popular design concept. It focuses on green energy saving, not letting resources waste, and protecting the natural environment. At present, cities in China have entered the stage of modernization. People can find that many cities are essentially the same except for the name of the city. These cities have lost their unique local atmosphere, and the buildings are dominated by monotonous tiles and glass. And these buildings consume a lot of energy. The more developed the urban economy, the greater the energy consumption of buildings. This will have a considerable impact on the local environment. It is precisely because these energy-intensive buildings obviously lack mutual communication with the natural environment, that some people put forward the concept of green design. It is hoped that the green building design space can be used to achieve the rational development of natural resources to reduce the resource consumption of buildings, so as to protect the ecological environment. However, in the green design of buildings, the adjustment of building space is always a problem. The human eye is always unable to estimate the distance and range of space very well. Therefore, in this regard, designers tend to be very detailed and spend a lot of time, and they can also avoid making mistakes in space adjustment.

The main function of the vision sensor is to obtain enough raw images to be processed by the machine vision system and then analyze them. It costs less and is very convenient to use. And now its development is very fast, and its application range is also very wide. Even if the image to be acquired is not very close, or in non-static mode, the sensor can make a good judgment. The innovation of this study is to use a different method, visual sensor image analysis, to conduct a strategic study on the construction of green building design space adjustment. During the research process, many simulation analyses were done on the adjustment of the design space with this sensor, trying to get the best strategy result.

Since the rise of green design in China, people have paid great attention to building energy efficiency, and more and more scholars have also done research on the construction of green building design. In recent years, Babu found that green buildings can significantly reduce or eliminate the negative impact of buildings on the environment, and can bring many environmental or resource benefits to human society [1]. However, he did not use relevant theoretical data to support his research content in the article. Lie et al. proposed a key technology for online virtual reality scene construction based on Virtual Reality Modeling Language (VRML) technology [2]. However, his data analysis summary in the article is not very good. Later, Xu proposed a green rural construction technology suitable for the northern region, and asked the technology to be considered from the perspective of saving resources [3]. However, the scope of the cases he analyzed in the article is not large enough, and it can only represent a part. Different from the research direction of other scholars, Arokiaprakash and Kumar tried to find out the various factors hindering the successful implementation of green buildings in the Indian construction industry through a comprehensive study of the literature [4]. However, the questionnaire survey he did in the article is not very comprehensive.

And there are many related researches on visual sensors. Wu selected two typical chips from two kinds of vision chips to study their structure and working mode [5]. But he did not use strong data to prove his argument in the article. Suárez et al. introduced a CMOS vision sensor chip using 0.18 *μ*m CMOS technology [6]. But when he compared the traditional and novel solutions, he ignored some factors that may have an impact. Later, Liu and Liu proposed a data fusion model for radar and vision pairs [7]. However, the model framework he proposed is too large and may not be able to achieve a convenient effect in reality.

## 2. Methods of Constructing Space Adjustment in Green Building Design

The content of this chapter mainly introduces the space adjustment of green building design and the related algorithms of visual sensor research. First, analyze what factors should be paid attention to when building space adjustment. Then, the algorithm of the related visual sensor is given, trying to find out the relationship between the two, so as to achieve the research purpose of this study.

### 2.1. Green Building Design Space Adjustment

The space adjustment of green building design is that architects use their professional knowledge to organize and design the building space reasonably, and create a moderate space to realize the indoor performance adjustment. Thereby improving the comfort of using the building and reducing the consumption of resources. With the proper spatial adjustment, buildings can consume no or less energy. This is very important for the design of green buildings [8]. The relationship between different buildings and ecological carrying capacity is also different, as shown in Figure 1.

As shown in Figure 1, the relationship between different buildings and ecological carrying capacity is also different. That is, different types of buildings have different impacts on the environment. Among them, ordinary buildings have the greatest impact on the environment, which has exceeded the ecological carrying capacity. That is to say, the energy consumption of the ordinary environment is very large, and it may cause irreparable damage to the environment for a long time. The impact of green buildings on the environment is precisely on the maximum ecological carrying capacity. That is to say, its impact on the environment is within the acceptable range of the ecological environment. It can effectively save energy and protect the environment. But there is another state of ideal architecture, which has the least impact on the environment, but it is still difficult to achieve such an ideal state. In short, it can be seen from the figure that green buildings are indeed much better than ordinary buildings in protecting the environment and saving resources, which is the main reason why the author chooses the theme of green buildings [9].

When designing space adjustments, in fact, the most important thing is to save energy, make reasonable use of available space and take care of the indoor environment. The layout of the space should start from the orientation of the building, the local climate, the received sunlight, lighting and natural ventilation [10].

Layout of the building: due to the concentration of buildings now, there are generally too many buildings in the area where the base is located or in the vicinity. There will also be an impact on lighting between buildings. If the layout of the base is not suitable, it is very likely that good sunlight conditions will not be obtained. However, if the buildings are arranged in a staggered and orderly manner, the shelters and gaps between them can be used, so that the buildings in the field can get appropriate sunlight [11], as shown in Figure 2.

From Figure 2, it can be found that if the houses are arranged in a staggered manner, the solar radiation received by the houses in the site can be averaged by using the gaps and occlusions between the walls. Some houses will not receive sunlight because the buildings on the side block are too much; and with a staggered arrangement, you can use the gable gap to increase the sunshine time. The combination of panel-type and point-type buildings can improve the sunlight effect [12].

Sunlight is especially important for constructing a building. The time limit that a house can accept sunlight will definitely affect the amount of solar radiation the house receives, so when building a house, pay attention to the natural lighting level of the house. And there are clear regulations in this area in China. Most cities require that the sunshine should not be less than 3 hours even in winter. As shown in Table 1, the real sun generally appears several tens of minutes earlier than the standard time. The azimuth and altitude of the sun are also different in different time periods. For example, when the standard time is 12 : 00, the actual time when the sun appears is actually 11 : 49. The azimuth angle is the largest in these time periods, at 176.8, and the altitude angle is also the largest in these time periods, at 37.9. It can be seen that the amount of solar radiation may be the most at 12 ‘o'clock. When building a house, considering the issue of sunlight, local solar data should also be referred to [13].

Ventilation treatment of buildings: as shown in Figure 3, the effect of several typical house layouts on ventilation can be clearly seen [14]. The determinant should be the most commonly used arrangement method for buildings at present, because it is arranged in rows and columns, and the houses are staggered before and after, so that the airflow can be inserted into the spacing. But the determinant has a relatively small wind surface in general. The staggered house layout because the houses are all facing the dominant wind direction in summer, staggered arrangement, increases the spacing of the houses, the wind can be introduced into the interior, and the distribution of the wind field is more reasonable. The inclined column layout can form a layout with small air inlets and large air outlets according to the wind direction, which can increase the flow rate of the wind and promote ventilation. Therefore, the ventilation effect of the staggered and oblique type is much better than that of the determinant, and it is suitable for many areas.

### 2.2. Algorithms for Vision Sensors

The human eye sees objects in three dimensions and can also estimate the distance of the objects seen [15]. However, human eyes are prone to visual deviation. The images seen by the eyes are transmitted to the human brain, and after processing, stereoscopic vision can be generated. This is the origin of stereo vision, as shown in Figure 4. Two eyes are two cameras, point *P* is a point to be tested. Because there are two cameras, one left and one right can get two points *P*_*l*_ and *P*_*r*_. Then, according to the known camera focal length *F* and baseline distance *B*, the coordinate value of *P* can be obtained through the principle of trigonometry. The formula for the depth difference can be expressed as

(1) $$\begin{array}{c} S=\left|P_{R}-P_{L}\right|\text{.} \end{array}$$

But there are some downsides to this measurement, as it does not have active light and does not work well in darker environments. It can only be used at close range, and the measurement error will be large in the distance [16].

Ranging principle: a vision sensor generally consists of an infrared camera and a transmitter, as shown in Figure 5. The transmitter projects an image to the object and the infrared camera receives the image reflected from the object.

It is an active measurement method, so it can be used in dark environments [17]. The measurement range of the structured light method is also relatively small, and it can only be measured at a close distance. Because the measurement distance will cause the reflected light to be very weak, the camera cannot recognize it. The principle of triangulation ranging is different from this, as shown in Figure 6. *S* is a lens, *N* is a projector, and *N* emits laser light to point *R* to form an image point *F* on the imaging surface. Because of the appearance of the occluding object *H*, the projector laser is emitted to point *H*, and a point *V* is left on the lens. The appearance of the occluded object *H* causes the laser imaging point to shift from point *F* to point *V*. The same laser beam changes with the depth of the irradiated object, and the image point formed on the imaging surface will shift. Then, people can know

(2) $$\begin{array}{c} VR:RG=f:J\text{.} \end{array}$$

Because VF is the offset and *J* is the distance from the camera to the object, we use *D* for depth; thus, we can say

(3) $$\begin{array}{c} RG:SN=\left(J-D\right):D\text{.} \end{array}$$

The distance between the camera and the transmitter is expressed as *K*, and the following formula can be obtained:

(4) $$\begin{array}{c} D=\frac{J*K*f}{K*f+H*∆Y}\text{,} \end{array}$$

(5) $$\begin{array}{c} ∆Y=M*O\text{.} \end{array}$$

*M* is the number of offset pixels, so the depth formula changes accordingly:

(6) $$\begin{array}{c} D=\frac{J*K*f}{K*f+H*M*O}\text{.} \end{array}$$

However, in actual shooting, the relationship between depth and offset is also very different [18]. As shown in Figure 7, according to our tests, it can be found that as the depth increases, the offset will decrease, and the greater the depth, the slower the offset will decrease. This means that the greater the depth, the greater the depth variation caused by each offset by one pixel, which will lead to an increase in the test depth and a decrease in the resolution of the system. So close-range tests are more accurate than long-range tests.

Learning algorithm: Learning algorithms are able to discriminate model predictions well. The error function is generally defined by least squares, and the formula is as follows:

(7) $$\begin{array}{c} K=\frac{1}{2}\overset{M}{\underset{H=1}{\sum }}{\left(Y_{K}^{F}-Y_{K}^{P}\right)}^{2}\text{,} \end{array}$$

where *Y*_*K*_^*F*^ refers to the time of laser release, and *Y*_*K*_^*P*^ is the actual release time. Then because of backpropagation people can get the following formula:

(8) $$\begin{array}{c} ∆E_{OL}^{L}=-\vartheta \frac{\sigma K}{E_{OL}^{L}}\text{.} \end{array}$$

The learning error is because of the difference between the target output and the actual output, so its formula is

(9) $$\begin{array}{c} R=\sum_{K=1}^{M}\left(1-U_{K}\right)\left(I_{K}-B_{THR}\right)+U_{K}\left(B_{THR}-I_{K}\right)\text{.} \end{array}$$

Among them, *I*_*K*_ is the maximum value, *U*_*K*_ is the actual category, and *U*_*K*_ can be expressed as

(10) $$\begin{array}{c} U_{K}=\left\{\begin{array}{cc} 1\text{,} & O=U\text{,}\\ 0\text{,} & O\neq U\text{.} \end{array}\right. \end{array}$$

Vision sensors generally capture static scenes, but when capturing dynamic scenes, the features are often the most abundant [19].

(11) $$\begin{array}{c} I\left(Y_{O}\right)=\underset{Y_{K}\leq Y_{O}}{\sum }L\left(Y_{O}-Y_{K}\right)+B_{REST}\text{,}\\ L\left(∆Y\right)=\text{EXP}\left(\frac{-∆Y}{\alpha_{N}}\right)\text{.} \end{array}$$

The moment when the laser transmission is dense is the moment when the information is the most abundant, and then the features are extracted, and then the formula can be obtained as

(12) $$\begin{array}{c} I_{YP}\geq I_{Y},\forall Y\in \left[Y_{P}-\frac{Y_{DT}}{2},Y_{P}+\frac{Y_{DT}}{2}\right]\text{.} \end{array}$$

Because of the occlusion of obstacles, the imaging will also be offset, the formula is as follows:

(13) $$\begin{array}{c} I\left(Y_{O}\right)=I\left(Y_{O}-1\right)\text{EXP}\left(-\frac{Y_{O}-Y_{O-1}}{Y}\right)+R_{O}\text{.} \end{array}$$

When in a two-dimensional plane, the sine and Gaussian functions of the camera and laser emitter can generate replica functions. *θ* is the angle of the camera and transmitter, and *τ* is the standard deviation of the distribution. Then, we can get the formula as follows:

(14) $$\begin{array}{c} H\left(C,U;\tau ,\rho ,\mu ,\tau \right)=\text{EXP}\left(-\frac{Y^{2}+X^{2}X^{2}}{2\beta^{2}}\right)\text{EXP}\left(O\left(2\pi \frac{Y}{\tau }+\varepsilon \right)\right)\text{,}\\ Y=XCOS\theta +USIN\theta \text{,}\\ X=-YSIN\theta +XCOS\theta \text{.} \end{array}$$

When identifying, if *μ*_*N*_ is the time constant, *B*_*REST*_ is the resting potential, and B is the membrane potential, the formula can be obtained as follows:

(15) $$\begin{array}{c} \mu_{N}\frac{FB}{FY}=B_{REST}-B+T_{N}O\left(Y\right)\text{.} \end{array}$$

If it is in the ideal state, the laser transmission is continuous, then the membrane potential of *Y* at any time can be obtained, as shown in the following formula:

(16) $$\begin{array}{c} B\left(Y\right)=\mu_{P}^{Y}OT_{M}R\frac{Y-C}{\vartheta M}=\vartheta MOT_{M}\left(1-R\frac{Y}{\vartheta M}\right)\text{.} \end{array}$$

Assuming that the threshold value is *B*_*YJ*_, then under the influence of a constant current *O*, the time consuming *Y* for *B*_*REST*_ to rise to the threshold value *B*_*YJ*_ can be expressed as the following formula:

(17) $$\begin{array}{c} Y=-\vartheta MLN\left(1-\frac{B_{YJ}-B_{REST}}{OT_{N}}\right)\text{.} \end{array}$$

## 3. Experiment and Deconstruction

The above part has analyzed the space adjustment and visual sensor of green building design. Therefore, this part will make a comprehensive survey and statistics on the status quo of domestic green buildings, study the current project situation. And find the connection between vision sensor and building space regulation. Finally, the performance advantages of visual sensors in constructing buildings for spatial adjustment are studied.

### 3.1. Deconstruction of the Status Quo

In fact, since the introduction of green buildings, the development of this aspect in China has been very fast [20]. Many projects are set up in this mode.  Figure 8 can be obtained according to relevant statistics. It can be seen from the figure that the number of projects belongs to a rising trend, and the development is very fast. But the project still has room to grow. Although the development of first-tier cities has been very stable because the development of second-tier and third-tier cities started slowly, a certain market has not been formed. In 2021, there are already 980 one-star projects, 1,040 two-star projects, and 850 Samsung projects. The development of Samsung is a little slower than that of one star and two stars, and the development of two stars is the fastest. Judging from the statistics, there should be more development in Samsung's projects.

After subdivision, a corresponding table can be made according to the number of projects and building area, as shown in Table 2. Because the country is too broad, people cannot do all the statistics and people can only study and investigate by sampling [21]. Therefore, people only selected five places for research. A lot of information can be obtained from the table. People can find that the Jiangsu area has the most projects, with 187 projects, which means that there are more green building projects in the more developed areas. The last place is Beijing, which has only 65, mainly because many state-protected buildings in Beijing cannot be easily changed. Then, regarding the construction area, it is also the largest in Jiangsu, with 18.99 million square meters, and Beijing with 5.3 million square meters. In short, the economic development of a city will still affect the number of green building projects in the area. And the impact is still huge. Therefore, if people want to build green buildings in an all-round way, you should vigorously improve the economic level of each region.

In the application of green building technology, the application of residential buildings and public buildings is also different [22]. As shown in Table 3, it can be clearly found that in the green lighting system, both residential buildings and public buildings use 100% of this technology. On the solar water heating system, the utilization rate of public buildings is 79%, and that of residential buildings is only 23%. It should be that residential buildings use other methods to heat hot water, such as gas water heaters, or electric water heaters. Therefore, the utilization rate of solar water heating systems in residential buildings is relatively low. In terms of high-efficiency HVAC systems, 95% of public buildings are used, compared to 59% of residential buildings. It may be because the population of public buildings is relatively concentrated, so this technology is generally used, while residential buildings belong to personal places and may not necessarily use this technology. On the intelligent system, the usage of both buildings is the same, both are 100%. On the rainwater recovery system, both buildings have the same utilization rate. This shows that the most unified part of the current construction application of this technology is the green lighting system and the intelligent system.

The weights of various evaluation indicators of green buildings are also very different, as shown in Table 4. There are a lot of evaluation indicators, and here we choose a more representative indicator [10]. It can be found that in the design stage and the operation stage, the indicator weights of the two types of buildings are biased. In the design stage, the energy saving of residential buildings is set at 0.25, and in the operation stage, it becomes 0.2, reducing the weight value. In terms of water saving, the public building is set to 0.19, and it becomes 0.15 in the operation stage, which also reduces the weight value. At the level of indoor environmental quality, in the design phase, residential buildings are 0.19 and public buildings are 0.2, but in the operation phase, the reductions are 0.15 and 0.16. This shows that in the actual operation stage, the weight value of each indicator will be reduced.

### 3.2. Experimental Deconstruction

Ranging algorithm experiment: after the above research on the current situation of domestic projects, it is further determined that the spatial adjustment can be analyzed by using visual sensors [23]. This study uses a case to demonstrate the feasibility and effectiveness of vision sensors in constructing space regulation in green building design. In order to better demonstrate the effect, people use the visual sensor to shoot different house space images at different measurement distances and use the ranging algorithm in this study to obtain the depth value of the image, as shown in Figure 9. It can be found that the house image obtained by close-up shooting is still very clear, and further architectural space adjustments can be made according to this three-dimensional image. The adjustment scheme obtained in this way is very accurate and reliable.

In order to ensure the accuracy of the test algorithm in this study, we also compare the test algorithm in this study with other algorithms, as shown in Figure 10.

As shown in Figure 10, the error of the ranging algorithm in this study is compared with other ranging algorithms under multiple measurement distances, where the red line refers to the ranging error of the ranging algorithm in this study. It can be seen intuitively from the figure that the error of the algorithm in this study in the measurement range of 1 m to 2 m is obviously smaller than that of other methods, and the accuracy is basically kept within 1 cm. The green lines indicate that the model is not very suitable for this study. The models with blue and red lines are relatively stable although they are controlled by error values. But the red line, that is, the algorithm model in this study, the obvious error value is smaller, and it will not affect the error value due to the change of distance. Finally, it is concluded that the error of the model will become very large as the distance increases, and its trend is an upward trend. There are two reasons for the low measurement error of the algorithm in this study: First, the ranging algorithm in this study finally obtains the depth value of each part in the image, and the final matching result of each part must be strictly screened. This makes the confidence of each part very high, and finally, the measured data has less noise. Second, after preprocessing by the local adaptive binarization method, the ranging algorithm can effectively deal with the changes of illumination and measurement background. In this study, the center pixel coordinates of each part are extracted, and the adjustment of the space often requires some control of the details, so the accuracy of the ranging algorithm in this study is high.

Thermal environment simulation: In order to explore the application performance advantages of vision sensors, we studied the specific relationship between the floor of the building's negative body and the thermal environment, and set up a simulation model experiment. Basic parameters of the model: the maximum square size of the building plane is set to 16.5 m∗16.5 m, the height is 9 m, the number of floors is 3, and the building facade is evenly opened with windows. Control the perimeter of the negative plane corresponding to the height of 4.5 m to 18 m, keep the window-to-wall ratio of each model consistent, the door size is 1.8 m∗2.1 m, and set the door opening directly to the south direction.

Set five basic models with negative body shape mouth-to-bottom ratios of 1 : 5, 1 : 3, 1 : 1, 3 : 1, and 5 : 1, respectively. For the negative shape of the rectangular section, a model with an aspect ratio *A* = 2 : 1 of the negative shape with an obvious thermal pressure ventilation mechanism was selected, and the thermal environment mechanism of the negative shape of the mouth-to-bottom ratio was discussed in detail. The solar radiation heat gain of each floor height of each model building is analyzed, including the direct heat gain and the diffuse heat gain. For the analysis height of each layer, divide the analysis grid, the grid precision is 100 × 100 mm. In the Ecotect calculation model, the detailed shading calculation is selected, and the accuracy of the sky is divided into fine 2′ × 2′(2 points *X* 2 points). The calculation time is set as June 22, and the calculation time is from 7 : 00 to 19 : 00 to realize the comprehensive calculation of effective radiation. Then use the visual sensor to identify and detect the simulated model. Finally, Figure 11 is obtained.

When the mouth-to-bottom ratio of the negative body is *B* = 1, with the increase of the mouth-to-bottom ratio B, the average radiation area of each layer gradually increases, and the increase is larger. When the negative body-shaped mouth-to-bottom ratio *B* < 1, with the decrease of the mouth-to-bottom ratio B, the direct radiation gradually decreases due to the occlusion of the A-shaped section. The existence of the inclined façade increases the scattered radiation. When *B* = 1 : 5, the scattered radiation gain cannot compensate for the loss of direct radiation. Therefore, the change trend of the average radiation area of each layer shows a gradual increase at first and then a gradual decrease, with a small increase and decrease. With the decrease of the mouth-to-bottom ratio B of the negative body shape, the broken line of the average radiation area tends to be flat, indicating that the radiation uniformity is gradually improved. In the simulation model with a negative body shape mouth-to-bottom ratio *B* < 1, the average radiation area decreases first and then increases with the increase of vertical height. While in the simulation model with negative body aspect ratio *B* > 1, the average radiation area increases with the increase of vertical height. Based on the above analysis, the following conclusions are drawn: When the negative shape of the cross-section is V-shaped, the larger the ratio of the mouth to the bottom of the negative body is, the greater the heat gain in the building. When the negative shape of the cross-section is A-shaped and the ratio of the mouth to the bottom of the negative shape is *B* = 1 : 3, the heat gain in the building is the largest. The smaller the negative body bottom ratio B, the better the indoor radiation uniformity of the building. When the ratio of the negative body to the bottom of the mouth is *B* > 1, the higher the vertical height, the better the heat gain. When the negative body shape mouth-to-bottom ratio *B* < 1, the heat gain first decreased and then increased with the increase of vertical height. These data are all obtained under the recognition mode of the visual sensor, it can be seen that this technology is very suitable for the spatial adjustment of green buildings.

In order to prove the merits of visual sensors in building space adjustment, we compared different network models, and the results are shown in Table 5. People can find that the performance of each visual sensor network model on buildings is also different. The first recognition tool can only barely guarantee the recognition effectiveness of a single class on buildings, and the recognition effect of other buildings with too many obstacles is poor. This is mainly because, in the training samples, each frame of data contains walls, which account for a large proportion of the training samples, so the network has a good effect on building recognition. For other categories with a relatively small proportion, the network fitting effect is relatively poor. After the second identification tool and the technology used in this study are added to the back-end optimization network, compared with the first tool, they still have a certain classification accuracy on the test set. Among them, the technology used in this study has the highest classification accuracy under the dual constraints of lidar high-precision information and image information. Therefore, it is concluded that vision sensors are very good at identifying buildings with accuracy.

## 4. Conclusion

In this study, the research and analysis of the construction strategy of constructing space adjustment in green building design are carried out through visual sensors, and it is concluded that the use of visual sensors is of great help to the development of space adjustment. Due to the current advocacy for green design, many factors need to be considered when designing buildings. Because these spatial influencing factors are likely to cause waste of resources, it is necessary to use external auxiliary tools, that is, visual sensors, to help architects obtain accurate data, so as to conduct scientific and accurate analysis of buildings. In general, the technology studied in this study is very suitable for use in the adjustment of green design space, and domestic research on visual sensors in green design should be increased. However, due to the limited space of the article, more influencing factors were not considered when studying the performance of the technology, so it could not cover all aspects. At the same time, there are not many examples used in this study, and only some regions are selected as the research objects, so the results may not represent macroscopic significance. This is also the limitation of this study. In the future, the author looks forward to using more real data to conduct in-depth research, so as to explore the research results of more visual sensors in the adjustment of green design space.

## Figures and Tables

**Figure 1:** Relationship between different buildings and ecological carrying capacity.

**Figure 2:** Influence of building layout on sunlight. (a) Staggered arrangement. (b) Plate point type.

**Figure 3:** Effect of building group layout on ventilation. (a) Determinant. (b) Staggered. (c) Inclined column.

**Figure 4:** Schematic diagram of stereo vision depth ranging.

**Figure 5:** Schematic diagram of structured light ranging.

**Figure 6:** Structured light ranging principle. ∆*Y* is the offset, which is for a camera with cell size *O*. (a) No obstructions. (b) Obstruction exists.

**Figure 7:** Depth vs. offset.

**Figure 8:** Status of green building development evaluation and identification projects.

**Figure 9:** 3D image obtained by ranging algorithm.

**Figure 10:** Algorithm comparison.

**Figure 11:** Line figure of radiation area. (a) Line graph of the average radiation area of each aspect ratio. (b) Line graph of the average radiation area of each layer.

**Table 1:** Sun data sheet.

Standard time	Standard time	Azimuth	High angle

08 : 00	07 : 49	122.2	10.5
10 : 00	09 : 49	144.6	29.2
12 : 00	11 : 49	176.8	37.9
14 : 00	13 : 49	−149.9	31.8
16 : 00	15 : 49	−125.7	14.4

**Table 2:** Geographical distribution of green building evaluation marks.

Region	The number of projects	Area of the building

Jiangsu	187	1899
Guangdong	103	945
Shanghai	89	659
Shandong	67	650
Beijing	65	530

**Table 3:** Statistics on the application of green building technology.

Technology	Residential building	Public buildings

Green lighting system	100%	100%
Solar water heating system	23%	79%
High-efficiency HVAC system	59%	95%
Intelligent system	100%	100%
Rainwater recovery system	68%	68%

**Table 4:** Weights of various evaluation indicators for green buildings.

A project phase	Building type	Save land and outdoor environment	Energy conservation and utilization	Water conservation and utilization	Material saving and material resource utilization	Indoor environmental quality

The design phase	Residential building	0.22	0.25	0.3	0.18	0.19
	Public buildings	0.17	0.29	0.19	0.2	0.2

Operation stages	Residential building	0.18	0.2	0.17	0.15	0.15
	Public buildings	0.14	0.24	0.15	0.16	0.16

**Table 5:** The performance of each network model on building recognition.

A network model	Average pixel accuracy %	The average IOU (%)	Average processing time (ms)

Identification tool 1	33.2	25.3	14
Identification tool 2	53.4	49.7	89
Visual sensor	61.1	54	118

## Data Availability

The data used to support the findings of this study are available from the author upon request.
